The article "Value of Multislice Spiral CT in Differential Diagnosis of Thick-Wall Gallbladder Carcinoma and Chronic Cholecystitis" was retracted in 2023. Reasons: unreliable results or conclusions; concerns about the data; concerns about the peer review; concerns about the citations.

# Value of Multislice Spiral CT in Differential Diagnosis of Thick-Wall Gallbladder Carcinoma and Chronic Cholecystitis

**DOI:** 10.1155/2022/5459779

**Published:** 2022-05-06

**Authors:** Hua Han, Jun Han

**Affiliations:** ^1^Department of Radiology, The Third Affiliated Hospital of Jinzhou Medical University, Jinzhou 121000, Liaoning, China; ^2^Department of Radiology, The Third Affiliated Hospital of Chongqing Medical University, Chongqing 401120, China

## Abstract

To summarize the value of multislice spiral CT (MSCT) in the differential diagnosis of thick-wall gallbladder carcinoma (TWGC) and chronic cholecystitis (CC), the clinical data of 36 patients with TWGC and 60 patients with chronic cholecystitis who were treated in our hospital from January 2017 to May 2021 were retrospectively analyzed, and the CT image features and diagnostic accuracy of the patients were summarized. Compared with the CC group, the proportions of disruption of gallbladder mucosa line, blurred gallbladder outline, high obstruction of biliary tract, lymphomegaly, adjacent invasion, peritoneal effusion, wall nodules, and the gallbladder wall thickness in the TWGC group were higher, with statistical significance (*P* < 0.05). Thirty-four patients with TWGC and 62 patients with chronic cholecystitis were diagnosed by MSCT. The sensitivity and specificity of MSCT in diagnosing TWGC were 86.11% and 95.00%, respectively. The positive likelihood ratio was 17.222 and the negative likelihood ratio was 0.1462. The positive prediction rate was 91.18%, the negative prediction rate was 91.94%, and the correct rate was 91.67%. MSCT can show the characteristic difference between TWGC and chronic cholecystitis, which can be used for differential diagnosis.

## 1. Introduction

As a common malignant tumor of the biliary system, gallbladder cancer can be divided into mass type, thick-walled type, and intraluminal type according to different imaging manifestations. Thick-wall gallbladder carcinoma (TWGC) accounts for 13%–25% of all gallbladder cancers [1]. It is difficult to distinguish TWGC from chronic cholecystitis due to lack of specificity in clinical symptoms and signs and overlapping imaging manifestations [2]. At present, ultrasound and abdominal CT are the conventional imaging methods for gallbladder cancer. With the update of imaging technology, the diagnostic level of gallbladder cancer has been improved significantly. However, it is still difficult to distinguish TWGC from chronic cholecystitis regardless of clinical diagnosis or imaging diagnosis [3]. Therefore, how to improve the differential diagnosis accuracy between TWGC and chronic cholecystitis is an urgent problem to be solved. Multislice spiral CT dual-phase enhanced scan can not only show the enhancement characteristics of the lesion but also has a significantly better inspection effect than B-ultrasound in the location and shape of the lesion, as well as the status of the affected lymph node and distant metastasis of adjacent liver tissues [4]. Currently, there are few studies on the application of MSCT in the differential diagnosis of TWGC and chronic cholecystitis. Therefore, in this study, MSCT images of 36 TWGC patients and 60 chronic cholecystitis patients were retrospectively analyzed in order to explore the imaging differences between TWGC and chronic cholecystitis in order to improve the clinical differential diagnosis ability.

## 2. Materials and Methods

### 2.1. Clinical Information

The clinical data of 36 patients with TWGC and 60 patients with chronic cholecystitis who were treated in our hospital from January 2017 to May 2021 were retrospectively analyzed. Inclusion criteria were as follows. (1) All patients' diseases were confirmed by pathological diagnosis. All patients conformed to the surgical and pathological results of thick-walled gallbladder carcinoma and chronic cholecystitis. (2) Hospital diagnosis and treatment, examination data, imaging examination reports, and other data are perfect. Exclusion criteria were as follows: younger than 18 years or older than 75 years, have a history of mental illness, and suffer from AIDS, tuberculosis, and other diseases. There were 96 patients in total, aged 35–76 years, with an average of (62.31 ± 6.64) years, who were selected for the study. Among TWGC patients, 28 were adenocarcinoma, 5 were squamous carcinoma, and 3 were undifferentiated carcinoma. There were 15 cases of right upper abdominal pain or discomfort and tenderness under the xiphoid process, 10 cases of skin and sclera yellow staining, 8 cases of upper abdominal touch mass, and 3 cases of emaciation and fatigue. Among the patients with chronic cholecystitis, 37 had cholecystolithiasis, 20 had no calculi, and 3 had xanthogranulomatous chronic cholecystitis. There were 46 cases of abdominal pain, fullness, and oil aversion, 9 cases of right shoulder pain, 3 cases of skin sclera yellow staining, and 2 cases of low fever. TWGC patients were enrolled in the TWGC group, and chronic cholecystitis patients were enrolled in the CC group. This study was approved by the medical ethics committee of our hospital, and both the subjects and the families signed the informed consent forms.

### 2.2. Methods

Preparation before examination: the patient fasted for more than 12 h, drank 300 mL isotonic mannitol every 15 min for 3 times to fill the intestinal tract, and then drank 300 mL isotonic mannitol for 4 times to fill the gastric cavity before going to the examination bed. Routine plain and enhanced hepatobiliary scans (from the top of the liver to the iliac crest) were performed in all patients using an Aquilion 128 layer CT scanner (Toshiba Company, Japan). The scanning methods were as follows: plain CT scan was performed first, followed by enhanced examination of arterial and portal veins. Arterial phase scan: the scanning was started 37 s after injection of a specific agent through the cubital vein of the upper limb. Portal vein phase scan: the scanning was started from 60 s to 70 s after contrast agent injection, and 3D recombination of plain and enhanced dual-phase scanning was performed. The scanning delay time is 5 minutes, 10 minutes, and 15 minutes. Set the scanning parameters as follows: voltage 120 kV, tube current 150 mA, thick layer 1.50 cm, and pitch 1.375 : 1. 100 mL contrast agent (Beilu Pharmaceutical Co., Ltd., Beijing, China) was injected under high pressure at a rate of 3.5 mL/s, and the scanning time was less than 5 s after 25 s delay. Bone function and soft tissue function were selected for the reconstructed images. The interval and reconstructed thicknesses were 1.0 mm and 1.5 mm, respectively. All parameters were sent to Vitrea 4.0 workstation for processing.

### 2.3. Observation Indicators and Evaluation Criteria

Analysis of MSCT images of all patients was performed by the same group of attending physicians and associate chief physicians. Gallbladder wall thickened: thickened more than 4 mm and uneven. Gallbladder wall stiffness: the gallbladder wall loses its normal outline, showing rigidity and irregular and incomplete shape. Interruption of the mucous line of the gallbladder: it is mainly characterized by the interruption of the mucous line of two or more layers. Gallbladder blurring: blurring or disappearance of fatty bands between the gallbladder and adjacent organs. Biliary obstruction: systemic dilation in the hepatic duct above the hilum was considered as high obstruction, while dilation in the lower common bile duct was considered as low obstruction. Invasion of the liver: liver gallbladder boundary is unclear, patchy low-density shadow in liver, and enhanced patchy enhancement. Lymph node enlargement: single lymph node diameter greater than 10 mm or multiple diameter greater than 7 mm. Small amount of peritoneal effusion: crescent-shaped, narrow band fluid low-density area around the liver, gallbladder, and spleen [5].

### 2.4. Statistical Methods

All collected data were input into EpiData V 3.1 database and analyzed in SAS 9.3 (SAS Institute Inc., Cary, NC, USA.). The inspection level is *α* = 0.05. All statistics are denoted by $\bar{x}\pm s$. The *t*-test was used to compare two groups, and the variance test was used to compare multiple groups. Categorical variables were expressed by rate or composition ratio and analyzed with the *χ*^2^ test. The kappa test was used for the consistency analysis. A *P* value <0.05 indicated that the difference was statistically significant.

## 3. Results

### 3.1. Differences in General Data

Compared with the CC group, the TWGC group showed no significant difference in gender distribution and average age (*P* > 0.05), as given in Table 1 and Figure 1.

### 3.2. Differences in Enhancement Features and MSCT Features

Characteristics of enhancement: in the TWGC group, the enhancement mode was high density of lesion site in arterial phase and isodensity of lesion site in portal vein phase. The enhancement pattern of the CC group was isodensity of lesion site in both arterial and portal phases.

Compared with the CC group, the proportions of cystic mucosa line disruption, gallbladder contour ambiguity, high biliary tract obstruction, lymphomegaly, adjacent invasion, hydrops abdominis, and mural nodules and the gallbladder wall thickness of the TWGC group were higher, with statistical significance (*P* < 0.05), as given in Table 2 and Figures 2–4.

The patient, a 74-year-old male, was diagnosed with TWGC. Multislice spiral CT showed that the tumor cells were columnar and varied in size, infiltrating the whole gallbladder wall, involving the entire gallbladder, invading nerves, and surrounding adipose tissue. Repeated atypical hyperplasia of the mucosal epithelium at the broken end did not invade the liver, and no cancer metastasis was observed in lymph nodes. The gallbladder wall was diffusely thickened, with a thickness of 0.8–1.5 cm, and no hard nodules were touched. There is a lymph node with a diameter of 0.2 cm.

The patient, a 37-year-old man, was diagnosed with chronic cholecystitis. MSCT showed rough gallbladder mucosa and 1.5 cm thick gallbladder wall. No nodule or mass was observed, and the mucosal line was intact.

### 3.3. Differential Diagnosis of TWGC and Chronic Cholecystitis by MSCT

Thirty-four patients with TWGC and 62 patients with chronic cholecystitis were diagnosed by MSCT. The sensitivity of MSCT in diagnosing TWGC was 86.11% (31/36) and the specificity was 95.00% (57/60). The positive likelihood ratio was 17.222 (86.11%/(1–95.00%)) and the negative likelihood ratio was 0.1462 ((1–86.11%)/95.00%). The positive prediction rate was 91.18% (31/34), the negative prediction rate was 91.94% (57/62), and the correct rate was 91.67% ((31 + 57)/96), as given in Table 3.

## 4. Discussion

Gallbladder cancer tends to occur at the bottom of the gallbladder body, and its pathogenesis is still unclear, which may be related to long-term exposure to carcinogens, abnormal biliary drainage, malignant transformation of benign gallbladder tumors, and chronic cholecystitis or stimulation of gallstones [6]. The onset of this disease is insidious, and its early symptoms are very similar to chronic cholecystitis. It is a difficult problem for clinicians to accurately identify these two diseases. Gallbladder cancer tends to occur in the elderly and is mostly female [7], which may be related to the high incidence of cholelithiasis and cholecystitis in elderly women. Spiral CT has high temporal resolution, spatial resolution, and density resolution and has a wide range of applications. It can complete large-scale scanning in a short time, get volume images, and reduce motion artifacts. The image quality is greatly improved compared with ordinary CT, so it can improve the accuracy of diagnosis [8]. Through imaging, it was found that the thickness of gallbladder wall in patients with thick-walled gallbladder carcinoma was larger, the gallbladder was blurred, and the gallbladder mucosal line was interrupted, high bile duct obstruction occurred more frequently, and it was easy to occur a small amount of fluid in the abdominal cavity, invasion of the liver, and enlargement of lymph nodes. In patients with chronic cholecystitis, the thickness of the gallbladder wall is small, the gallbladder is clearly visible, and the gallbladder mucosal line is intact; lower bile duct obstruction occurs more frequently, and there is no small amount of abdominal effusion, liver invasion, and lymph node enlargement. Therefore, spiral CT can clearly distinguish the two diseases and lay the foundation for follow-up treatment [9].

The results of this study showed that TWGC patients often had damaged and interrupted cystic mucosa line, blurred gallbladder outline, and high obstruction of the biliary tract, and there was a high proportion of lymphadenopathy, adjacent invasion, and hydrops abdominis, while there was no lymphadenopathy, adjacent invasion, and hydrops abdominis in patients with chronic cholecystitis. Cystic mucosa line is the continuous smooth and dense circular line shadow of capillaries in the inner wall of the gallbladder under CT scan [10]. The cancer cells of gallbladder cancer invade the structures of each layer of the cystic wall, resulting in the erosion and destruction of capillaries of the proper layer of the cystic wall. Therefore, enhanced CT scan of TWGC patients showed that the cystic mucosa line was interrupted, showing discontinuous nonclosed rings [11]. In general, chronic cholecystitis rarely damages the lamina propria, so the gallbladder mucosa is often continuous and complete, and the enhanced scan mucosa presents annular enhancement [12]. TWGC is a malignant lesion, and cancer cells in patients can easily penetrate through the muscularum to the serosa, thus invading the adipose tissue and adjacent liver tissue in the gallbladder fossa, resulting in blurred gallbladder outline [8]. However, chronic cholecystitis is a benign disease with limitations on surrounding liver infiltration, so the hepatobiliary interface of most patients still exists and the gallbladder is clearly defined [13]. Bile duct dilation is an indirect sign of gallbladder cancer, which is triggered by bile duct compression, tumor invasion of the common bile duct, and tumor spread through the bile duct [14]. Low biliary tract obstruction is caused by bile duct dilation causing stones to enter the lower common bile duct, and high biliary tract obstruction is caused by Mirizzi syndrome [15, 16]. Patients with chronic cholecystitis are less likely to have high or low obstruction because of the absence of bile duct dilation. The metastasis pathways of gallbladder cancer include direct invasion, lymph node metastasis, hematogenous metastasis, intrabile duct metastasis, and peritoneal implantation, among which direct invasion of adjacent normal tissues and organs and lymph node metastasis are the most common [17, 18]. In this study, there were 13 patients with TWGC, accounting for 36.11%. In the results of this study, the gallbladder wall thickness in TWGC patients was over 9.5 mm on average, which was significantly thicker than that in patients with chronic cholecystitis. The normal range of gallbladder wall thickness for adults is ≤3.0 mm, and thickening beyond this range is considered [19]. Both TWGC and chronic cholecystitis can cause gallbladder wall thickening, but the morphology of gallbladder wall thickening caused by TWGC and chronic cholecystitis is obviously different. Among them, the gallbladder wall of TWGC is mainly thickened with local irregularities, while the cystic wall of chronic cholecystitis is generally thickened with extensive and uniform consistency, and the inner wall of the cystic wall is relatively smooth. Compared with chronic cholecystitis, TWGC is more prone to mural nodules. The study also found that the proportion of TWGC patients with mural nodules was 52.78%, which was significantly higher than 15% of chronic cholecystitis. In TWGC patients, the enhancement mode was high density of lesion site in arterial phase and isodensity of lesion site in portal vein phase. The enhancement mode of CC patients was isodensity of lesion site in both arterial phase and portal vein phase. Therefore, the degree and mode of enhancement in arterial and portal phases of gallbladder cancer are different, which is helpful to distinguish TWGC from chronic cholecystitis.

## 5. Conclusion

The clinical manifestations of chronic cholecystitis and thick-walled gallbladder carcinoma are the same, including right abdominal pain and jaundice. It is easy to misdiagnose, confuse, and delay the patient's condition in diagnosis, so it is of great value to distinguish between the two diseases. Spiral CT can clearly distinguish the two diseases with high accuracy, which can be used as a basis for clinical diagnosis and differentiation of chronic cholecystitis and thick-walled gallbladder cancer, provide reliable data for later treatment, and can be widely used in clinical diagnosis.

## Figures and Tables

**Figure 1:** Differences in general data. (a) Gender. (b) age. Compared with the CC group, the TWGC group showed no significant difference in gender distribution and average age (*P* > 0.05).

**Figure 2:** Differences in the characteristics of MSCT. (a) Cystic mucosa line. (b) Gallbladder outline. (c) Biliary infarction. (d) Gallbladder wall thickness. (e) Mural nodules. Compared with the CC group, the proportions of cystic mucosa line disruption, gallbladder contour ambiguity, high biliary tract obstruction, lymphomegaly, adjacent invasion, hydrops abdominis, and mural nodules and the gallbladder wall thickness of the TWGC group were higher, with statistical significance (*P* < 0.05).

**Figure 3:** MSCT examination of TWGC patients.

**Figure 4:** MSCT examination of chronic cholecystitis.

**Table 1:** Differences in general data.

CT signal	Gender (*n* (%), case)		Age ($\bar{x}\pm s$, year)
	Female	Male	
TWGCG group (*n* = 36)	29 (80.56)	7 (19.44)	61.28 ± 6.24
CC group (*n* = 60)	44 (73.33)	16 (26.67)	63.34 ± 7.04
*χ* ^2^ */t*	0.644		1.447
*P*	0.422		0.151

**Table 2:** Differences in the characteristics of MSCT.

CT signal	TWGC group (*n* = 36)	CC group (*n* = 60)	*t*/*χ*^2^	*P*
Cystic mucosa line (*n* (%), case)			65.336	<0.001
Interrupt	33 (91.67)	5 (8.33)		
Intactness	3 (8.33)	55 (91.67)		
Gallbladder outline (*n* (%), case)			43.556	<0.001
Fuzzy	30 (83.33)	9 (15.00)		
Clear	6 (16.67)	51 (85.00)		
Biliary infarction (*n* (%), case)			−3.792	<0.001
High-order position	9 (25.00)	1 (1.67)		
Low-order position	2 (5.56)	1 (1.67)		
Without	25 (69.44)	58 (96.67)		
Lymphadenectasis (*n* (%), case)			48.793	<0.001
With	20 (55.56)	0 (0)		
Without	16 (44.44)	60 (100.00)		
Adjacent invasion (*n* (%), case)				
With	13 (36.11)	0 (0)	29.047	<0.001
Without	23 (63.89)	60 (100.00)		
Hydrops abdominis (*n* (%), case)			10.272	0.001
With	5 (13.89)	0 (0)		
Without	31 (86.11)	60 (100.00)		
Gallbladder wall thickness ($\bar{x}\pm s$, mm)	9.85 ± 1.52	7.53 ± 2.04	5.906	<0.001
Mural nodules (*n* (%), case)			15.543	<0.001
With	19 (52.78)	9 (15.00)		
Without	17 (47.22)	51 (85.00)		

**Table 3:** Differential diagnosis of TWGC and chronic cholecystitis by MSCT.

CT diagnosis	Pathological diagnosis		Total
	TWGC (36 cases)	Chronic cholecystitis (60 cases)	
TWGC	31	3 (misdiagnose)	34
Chronic cholecystitis	5 (misdiagnose)	57	62
Total	36	60	96

## Data Availability

The simulation experiment data used to support the findings of this study are available from the corresponding author upon request.
